# Design of a Multimedia-Assisted Distance English Teaching System for College Students

**DOI:** 10.1155/2022/2184600

**Published:** 2022-06-16

**Authors:** Haili Feng

**Affiliations:** School of Foreign Languages, Qiongtai Normal University, Haikou 571127, China

## Abstract

To address the problems of poor compatibility, weak load capacity, and time consumption of existing multimedia-assisted teaching systems, we propose and design a physics multimedia-assisted English teaching system based on a concept network. The architecture of the physics multimedia-assisted teaching system is constructed with the logical layer as the core, and the theoretical knowledge module, experiment module, and student practice module are designed, respectively. Based on the concept network, a large number of rules in the physics teaching system are attached to the concepts to form the concept network knowledge system and complete the design of the theoretical knowledge system. This paper explores the multimedia teaching of college English and points out the advantages and characteristics of this teaching mode and the problems to be paid attention to in the process of application. The design of the physics multimedia-assisted teaching system is completed by realizing students' practice and giving feedback on the practice results. The experimental results show that the system has good compatibility, strong load capacity, low time consumption, and practical application value.

## 1. Introduction

University education, an important part of the national higher education system, has been developing rapidly in China in recent years. In order to promote the vigorous development of university education and meet the needs of social and economic development, the Ministry of Education has been actively promoting the reform of university education, and the reform of university English courses also needs to meet the needs of the times [1, 2]. The rapid development of information technology and the increasing maturity of computer network technology have made education more and more modernized, and the application of multimedia technology is one of the important symbols of education modernization [3, 4]. Multimedia teaching is the latest stage of development of modern English teaching, which provides a colorful expression for English teaching with the characteristics of large amount of information, fast transmission, graphic and text, human-computer dialogue, clear interface, effective combination of audio-visual, convenient information retrieval and high efficiency, and so on [5]. It injects new colors and vitality into the classroom and is becoming more and more important in English teaching [6].

Multimedia-assisted English teaching is conducive to giving full play to students' initiative and enthusiasm. Multimedia technology can make teaching forms more lively, further improve the quality of teaching, and change the passive acceptance of information to active acceptance of information, thus stimulating students' initiative and creativity [7]. Multimedia teaching integrates sound, image, video, and text, which can produce a lively effect and help improve students' interest in learning and memory ability [8]. It is better than the traditional teaching mode-textbook, chalk, or blackboard to stimulate students' learning enthusiasm [9]. Computer multimedia will be vivid images, vivid colors, and rich language and cultural scenes real in front of the students, and multimedia courseware with its images, graphics, text, sound, animation, and so on, a variety of functions on the students' multiple senses, can stimulate students' interest in learning, attract students' attention, more mobilize students' enthusiasm for learning, stimulate students' desire to learn, and give full play to students [10]. It is not only stimulating students' interest in learning and attracting their attention but also stimulating their enthusiasm for learning, stimulating their desire to learn, and giving full play to their initiative and enthusiasm [11].

It is also conducive to improving teaching efficiency and expanding classroom capacity [12]. Multimedia-assisted English teaching can expand the amount of classroom information, make full use of classroom teaching time, greatly enrich and improve the content of foreign language teaching, and fundamentally improve teaching efficiency [13, 14]. Teachers and students can use the information resources stored on CDs, VCDs, floppy disks, CD-ROMs, and hard disks in the multimedia classroom and can also use multimedia courseware for teaching, which can create a vivid, imaginative, authentic, and interesting English language environment for students, which is conducive to their understanding and mastery of teaching contents [15]. In traditional English classroom teaching, teachers spend most of the time on writing and explaining in each lesson, which is less dense and less informative, but teachers can increase the information of each lesson by arranging the board with the courseware, which can save time and make students get more knowledge in the same time and improve the learning efficiency [16, 17].

The use of multimedia technology in teaching puts forward higher requirements for teachers, who should not only know educational technology and teaching theory and have a high level of English but also have a certain ability to use computers [18]. Through multimedia courseware, teachers can design a new teaching process, display subtle teaching ideas and new creativity, expand the capacity of classroom teaching, and attract students' pursuit of knowledge, which is both promotion and challenge for teachers and a process of improving themselves. Multimedia teaching can also effectively use network resources [19]. There is a large amount of information related to English teaching content on the Internet, so teachers can use the Internet to download the content they need and expand the language materials so that students can use and obtain the latest information. This not only enriches the teaching content dynamically but also keeps the teachers' teaching ideas and content up to date with the development of the times [20].

## 2. System Design Principles and Functional Design

### 2.1. System Design Follows the Principles

The proposed English teaching system follows the following principles to carry out design: (1) Having complete functions: nowadays, most R&D enterprises are developing toward the level of intensification and scale, and according to the infrastructure and technology already available, all levels are closely united using information flow to achieve the purpose of unified management and data acquisition. (2) Modularity: the English teaching system is designed according to the principle of “modularity,” and the configuration is carried out according to the actual requirements of users, with relatively simple and flexible structured functional modules installed, and all basic and business modules can be combined at will to meet the existing or future system personalized application requirements. (3) Friendly operation interface: the design of a friendly and easy-to-operate interface helps users carry out the functions of each link, thus enhancing the efficiency of the system. The designed information input interface should follow the requirements of simplifying the actual work of users as much as possible and effectively reducing the error rate of data input. Therefore, in the process of designing this English teaching system, the user's memory burden should be reduced as much as possible, and automatic data input should be increased to avoid the situation of user data input errors. (4) High efficiency: the designed system should have high security and operation efficiency so as to provide users with high-quality services and obtain a quick response and relatively stable system. In addition, each program and interface of the system must be designed with a uniform standard to ensure that the system shows good portability and also facilitates timely expansion and application.

### 2.2. Overall System Architecture

Although the rapid development of computer and network technology has solved many problems, it is still a difficult problem to design and develop an English teaching system with complex information, such as how to secure the front-end of the system. The system architecture is the basis for the proper operation of a system, and its layout directly affects the stability of the system's operation. In the J2EE system, the server-side Web application is divided into several layers. Each of these layers is configured with significantly different functions and promises to be linked to different communication interfaces. The specific architecture of the system is shown in Figure 1.

In Figure 1, the JSP page is seen as the view layer, the main function of which is to smoothly implement the interaction between the system and the user and to display the final interaction combination directly using the JSP page. The view does not unfold the actual business but can accept data update operations so that the system interface can be updated at any time. Action control layer aims to receive response requests from the client user at any time and timely invoke the model in the business layer to smoothly realize the delivery of user requests. If the user submits a request using the page, mainly by sending an HTML form, the controller must respond to the request and finally deliver the result to the user using the view method. In one layer, the controller is implemented mainly through Action, ActionServlet, where Action can be called the corresponding adapter and separates the request from the business logic, thus combining the user's needs and calling the corresponding business logic components in time. The service business layer is located between the persistence layer and the Action layer, which is designed to implement the application logic and check the business, such as login password authentication. The main function of the DAO layer is to smoothly connect with the database, and the main function of the DAO layer is to smoothly connect to the database and perform various operations on the database, such as adding, modifying, deleting, and other business functions, but in J2EE development, SQL statements are generally used to smoothly implement the query operations, so that different interfaces can be called to achieve the corresponding functions.

### 2.3. Design of Each Function of the System

In order to improve the efficiency and level of students' learning English and to solve the time of learning English to a certain extent, the English teaching system designed in this study is based on advanced computer network technology, which is realized through the combination of J2EE, MVC architecture, and other technologies with related business, so that students can learn related services through this system and ensure that students can learn English audio materials, video materials, and so on at the first time. The system is designed to ensure that students have the first access to English audio and video materials. Based on this, combined with the actual needs of English teaching, the system functions are divided into the following functional modules in the paper, as shown in Figure 2.

In Figure 2, the authority management mainly consists of user login, user logout, user management, and other functions. To ensure more convenient system operation, the designed system login interface retains some similarities for different roles, and only some visual differences exist. After users enter their account numbers and passwords, the system automatically determines the user's identity type and quickly opens the operation privileges for that type of user. At the same time, the rights management is used to guide users to register on the website and for registered users to log in; the managerial rights include functions such as classification of user rights and user passwords. The teaching resource check includes two functions of joint and category search, with the help of which the required resource information can be searched according to the actual needs of users and the results can be directly linked to English teaching information. English audio/video on demand aims to realize the playback of English teaching videos or audios, and users can realize the download of English teaching resources with the help of this module. The resource management is mainly in the audio/video data uploading, deleting, and other operations to meet the needs of learners. The navigation management module is to meet the actual classification needs of the system. With the help of this function module, users can locate the required search resources in a very short time and start the operation of function switching and information finding according to the default order of the classification navigation configuration.

## 3. System Development Environment and Its Implementation

### 3.1. System Development Environment

In this study, RealNetworkHelixServer was selected as the streaming media server, which can support different formats, and the server supports some of the current mainstream playback software to better meet the needs of users. The operating system of the system is Win7, the development platform is My Eclipse 3.5, the server used is 70mcat6.5, the development technology is Struts2, Spring3, and Hibernate3, the configuration of MySQL5.0 database has the advantages of simple and easy to learn, the style of programming language is uniform, and the functions can be completed simply by using a few words. The SQL language is unified, simple, and easy to learn, all functions can be realized by combining a few English words, and this standardization makes it show its unique advantages in data storage and update.

### 3.2. Implementation of System Functions

#### 3.2.1. User Login Implementation

When designing the system login interface, the designers and developers generally use two security technologies to ensure the stability of the system and its safe operation. When users enter their own accounts and passwords, the user accounts and permissions are judged by the system code, and only when the visitors enter the correct accounts and passwords can they successfully enter the system to complete various operations. If the system suggests that the user has entered an incorrect account number or password, the system will restrict the visitor's access to the system and warn the illegal visitor in an appropriate way.

#### 3.2.2. Implementation of Third-Party Insertion Operation

In this paper, we would like to play the English audio/video material smoothly by inserting the corresponding player in the interface. Therefore, in the development process, we chose the ActiveX control technology, which is based on the principle of inserting an ActiveX control into the HTML file by using the object tag and accessing this space smoothly by using JavaScript.

### 3.3. Analysis of Application Examples

With the rapid development of computer technology, nowadays, most of the new resources for teaching English in schools are saved in the form of audio and video, which requires higher requirements in terms of real-time transmission and certain quality assurance; RTP/RTCP can provide real-time transmission control services for streaming media and has QoS to ensure that the purpose of teaching resources transmission can be achieved through this protocol. RTP/RTCP real-time video transmission can be based on compression coding to collect English teaching video to perform compression coding operations; the most basic process includes video capture, encoding, decoding, and other operations, as shown in Figure 3.

On the server side, the collected audio and video information is used to generate the corresponding data source through compression coding. If a user requests access to the data information, the server receives the request information, generates a transmission channel at both the client and server endpoints, and then encapsulates the data source information in RTP packets to meet the actual needs of the client. At the same time, the RTCP feedback information is used to monitor the packet loss rate and the quality of service [21, 22].

## 4. Teaching System Architecture

Multimedia technology is based on animation, image, and other technologies as the core, and the content involves many fields such as communication, communication, and education. The multimedia-assisted teaching system is a new teaching method designed based on multimedia technology, which includes computer host, input/output devices, storage devices, and logic layer. The system architecture is shown in Figure 4.

In this paper, the logic layer is the core of the system design. Only by ensuring the smooth operation of the theoretical knowledge module, experiment module, and student practice module in the logic layer can the purpose of teaching system design be effectively realized. In this paper, the system design takes the teaching of the inaccuracy relationship in quantum mechanics as an example, and the specific module design is as follows.

### 4.1. Theoretical Knowledge Module Based on Conceptual Network

Conceptual network is an exploration of artificial intelligence research, using concepts as the basic nodes for describing objective things and the knowledge representation framework system of the association between things. Conceptual networks can integrate cognition, understanding, reasoning, and behavior into a whole and are used to guide the judgment and processing of intelligent systems for expected behaviors. A conceptual network consists of three elements: attributes, behaviors, and relationships [23, 24]. Attributes are inherent properties of things, behaviors are used to distinguish conceptual networks from other networks, and relationships are simple or complex associations formed between concepts. Conceptual network can produce a rule reasoning process, which is used to reflect the behavior of different concepts, so that a large number of rules in the physics teaching system can be attached to the knowledge system construction framework formed by the conceptual network, different things in different fields can form different knowledge systems based on their own characteristics and at the same time based on the framework, and this knowledge system construction method is more in line with the human thinking mode. The conceptual network is applied to the theoretical knowledge module to form the theoretical knowledge system, as shown in Figure 5.

### 4.2. Experimental Module

The teaching of the inaccuracy relationship of quantum mechanics includes the experiments of electron single slit diffraction, diffraction influencing factors, and the study of the number of incident particles. The experiments for variables such as single slit width are done by scrolling bars, and through the experimental settings, it is possible to apply the theoretical knowledge to reality and clearly show the particle diffraction streaks and the curve distribution using images and animations. The image design includes wave function and probability distribution diagram. The animation is an image that is dynamically displayed on the computer with regularity, and the animation is designed with a strong sense of realism, which can increase the interest in teaching. The images and animations formed in the experimental module design are realized through computer programming [25].

### 4.3. Student Practice Module

The design of the multimedia-assisted teaching system needs to incorporate the student-oriented education idea advocated in the current education field, which is a sign of educational progress and the basis for promoting the development of multimedia-assisted teaching. Based on the theoretical knowledge and experimental module mentioned above, student knowledge is modeled to ensure that student knowledge is consistent with theoretical knowledge and experimental knowledge, and student knowledge is compared with the theoretical knowledge system to form a comparison model, as shown in Figure 6.

In Figure 6, a value of 1 is assigned to each attribute node of the knowledge domain, and a range of values [0, 1] is also set in the student knowledge model. 0 means that the student has no knowledge at all, and 1 means that the student has completely mastered the knowledge of the node. In the initial stage of model construction, the values in the student model are set to 0. The student practice module is designed with several multiple-choice questions to complete the student practice based on the above mechanism and obtain the student behavior. Comprehensive analysis of the above modules can complete the design of multimedia-assisted teaching system of physics based on the concept network, as shown in Figure 7.

## 5. Experimental Results and Analysis

In order to test the performance of this system and conduct experimental analysis, the hardware configuration required for the operation of this system is 64 GB of internal memory, 256-color graphics card, 125 MB hard disk, and a monitor resolution of 1,024 × 768 pixels. The software configuration required for system operation is Windows XP operating system, data access component is MDAC2.8, and .Net Framework version 2.0 is used for the running environment. The system design is based on the Struts framework, which uses Servlet and JSP technology and has the function of unifying data resources, which can greatly save development time.

In the experimental analysis, 1 million data in the SQL Server database are selected as the data source, of which 500,000 data are used for system training and 500,000 data are used for system testing. The following experimental indexes are selected for experimental validation analysis: system load test and system time consumption.

### 5.1. Experiment 1

For a complete system, the load capacity size is a direct factor to determine the system performance, this experiment uses Web Application Stress for system load test, and the test parameters settings are shown in Table 1.

The test results were compared with literature [5, 7], and the results are shown in Figure 8.

Analysis of Figure 8 shows that no matter how the number of concurrent users changes, the system load rate of this paper is always lower than that of literature [5] and literature [6], and the low load rate means that the system can keep running efficiently for a longer time, which indicates that the system of this paper has better load capacity and is better than other literature methods.

### 5.2. Experiment 2

The running time of the system in this paper is compared with the systems in literature [5] and literature [7], and the results are shown in Figure 9.

From Figure 9, it can be seen that, with the increase in the amount of test data, the running time of the system in this paper shows a small increase, with the maximum time consumed being 15 s. The curves of literature [5] and literature [6] have a larger change and are more time-consuming, with a maximum value of 35 s, which is larger than the system in this paper. The low running time consumption and the significant advantage of the system in this paper are due to the fact that this paper uses conceptual networks to construct theoretical knowledge models and forms a knowledge representation framework, and the construction of this framework structure greatly reduces the complexity of model construction and saves time.

The use of computer-assisted multimedia teaching systems has provided us with great convenience in this area. Its role is to apply modern technology to stimulate and motivate students to think, to inspire their thinking, and to cultivate their ability to find, think, and solve problems. Due to the inertia of thinking, when we use multimedia-assisted teaching, most of the courseware is still stuck in only using the computer to show the phenomenon and impart knowledge, and many of them simply copy and electronize the textbook knowledge. As shown in Figure 10, teachers do not leave enough time for thinking, do not teach in a heuristic way, and show students all through multimedia, which will kill students' ability of independent learning and thinking over time. Therefore, when we design the courseware, we should start by improving students' ability and creating problem situations as much as possible to stimulate students' thinking so as to accelerate students' development. In multimedia-assisted English teaching, if we can pay attention to these problems, use the multimedia teaching system reasonably, create the situation of learning English, and let the advanced modern tools for teaching services so that students can perceive the English language materials through audio-visual.

## 6. Conclusion

Multimedia-assisted teaching system is a new mode of modern teaching, which can help teachers teach and assist students in completing independent learning. This paper designs a multimedia teaching system based on the concept network. The system design is completed by describing the theoretical knowledge module, experiment module, and student practice module based on the concept network. And the good performance of the system is verified through experiments, which has a certain reference value. However, there are still some shortcomings in the system design, and the interactive performance between students and teachers is not analyzed. In the subsequent research, we will focus on the analysis of the interactivity and further improve the system performance.

## Figures and Tables

**Figure 1:** Functional design of English teaching system.

**Figure 2:** Overall architecture of English teaching system.

**Figure 3:** Real-time video transmission operation.

**Figure 4:** Architecture of physics multimedia-assisted teaching system.

**Figure 5:** Conceptual network theory knowledge system.

**Figure 6:** Comparison of student knowledge and theoretical knowledge system.

**Figure 7:** Block diagram of multimedia-assisted teaching of physics.

**Figure 8:** Comparison of system load test results.

**Figure 9:** Comparison of system running time.

**Figure 10:** Effect of teaching English with different media.

**Table 1:** System load test parameters.

Test parameters	Numerical value
Test tools	Web application stress
Number of concurrent users	7
Running time (S)	5
Line type	Ethernet

## Data Availability

The experimental data used to support the findings of this study are available from the corresponding author upon request.
